# Construction of Internet Business Innovation Network Model and Data Image Research under the Background of Game Theory

**DOI:** 10.1155/2022/8804272

**Published:** 2022-01-06

**Authors:** Haiying Bai

**Affiliations:** Shanxi Forestry Vocational Technical College, Taiyuan, Shanxi 030009, China

## Abstract

Facing the fierce market competition, enterprises not only need a deeper understanding and concept renewal in marketing theory but also need a set of standardized, practical, and efficient technical means and methods. Therefore, it is urgent to develop advanced marketing analysis tools and marketing decision-making methods. Based on game theory and neural network model, this study simplifies the existing research methods. By introducing different models, an image analysis and decision-making model based on game theory and neural network is constructed. It mainly aims at enterprise decision-making. The method used is to simulate various decision-making processes of enterprises by establishing neural network model and game model. At the same time, the image simulation of the model is carried out. The results show that the highest market share of the selected products is 36.1%, and the highest brand awareness is 9 points. The product with the second market share has better quality, 8 brand awareness points, and the highest dealer fee (2.3 yuan). Market share is less affected by product price and dealer expenses. The accuracy of the designed market share neural network model is 93%. This shows that the increase of market share is not realized simply by reducing the price but by increasing the profits of distributors and improving the brand image. Market leaders have the greatest revenue and profits. There is a positive correlation between the efforts of managers and the results achieved. Internet employees' work effort is positively correlated with their basic salary. Different decisions have different effects on business models. The research of this paper provides a new idea for the innovation and development of Internet enterprise business model.

## 1. Introduction

At present, China is in the stage of rapid economic development in various fields, and the competition among enterprises is becoming increasingly fierce. Some scholars point out that the competition between social enterprises is the competition between business models [1]. Business model is one of the important research objects in the field of management. It is a kind of connection and transaction relationship between enterprises, between enterprises and customers, and between various departments within enterprises. It is the way, tool, and method for enterprises to create value, compete for consumers, occupy competitive advantage, and realize profits [2]. In addition, the business model is the cornerstone of the company's stable operation. Under the premise of rapid economic development, only by constantly innovating business models can enterprises add power to their own development [3]. In the new era, the Internet is developing rapidly, and the scale of China's Internet enterprises is huge. With its high efficiency and practical characteristics, the Internet provides a certain development opportunity for business model innovation. The research on business model innovation of Internet enterprises is one of the current hotspots [4].

It is mainly divided into strategic research, operations research, economic research, and integration research under the background of big data. Different research fields have different research methods, and there are many research methods of commercial enterprise innovation. Some studies show that the technology can be used to build information networks to enhance the flexibility of enterprises. In other image analysis studies, a theoretical model between business model, social capital, and absorptive capacity is established to discuss the innovation of business model [5]. With the development of neural network, it has been applied to the innovation of enterprise business model, which greatly simplifies the problem [6]. The neural network image analysis model is used to study the business model innovation of Internet enterprises, and the game theory is introduced to increase the analysis of the strategies of all parties in the business model. Game theory is a kind of decision-making behavior of rational decision-makers based on the study of the interaction of various strategies. It is widely used in many disciplines. The four elements of game theory are strategic space, participants in the game, participants' interests, and game order. The combination of game theory and neural network provides theoretical data guidance for the implementation of future strategic decision-making.

In the existing research, there is less research on the business model innovation of Internet enterprises under the neural network image analysis model, but the introduction of neural network and game theory has certain guiding significance for the business model innovation reform of Internet enterprises. Therefore, based on the review of relevant research and theoretical knowledge, the neural network model and game model are constructed. Finally, the model is simulated based on the actual data of Internet enterprises, and the quantitative experimental results are obtained. The innovation of this study is that the neural network model is applied to the business model innovation of Internet enterprises for the first time, which has important reference significance for the development of enterprise business model innovation.

## 2. Review and Analysis of Related Research

The concept of business model was proposed in the late 1950s. Liu and Jin summarized massive studies on the business model of scientists and analyzed the influencing factors of business model from various perspectives [7]. Hesser et al. found that the influencing factors of the business model include environmental analysis, stakeholders, corporate governance, competitive advantage, entrepreneur leadership, and objective mission. The direction and structure of the business model were mainly analyzed [8]. Dai et al. built the business model from the perspective of business ecology. The elements of the model included target customers, business systems, strategic positioning, and partners [9]. The research on business model innovation is mainly on the innovation driving force, including the decision-making ability of the executives and the overall level of the enterprise technology. Dong et al. found that the decision-making of enterprise executives plays a crucial role in the innovation of business model, and some studies made clear that enterprise technology exerts a fundamental impact on business model innovation [10]. Premananda et al. evaluated the overall level of enterprises and found that the four elements of the business model need to be integrated for effective innovation: core resources, value proposition, profit model, and important process [11].

The main direction of big data research based on business model innovation is the research on the business value of big data. Selma et al. established the business model based on that. The model shows great advantages in decision validation and data availability [12]. Kao and Venkatachalam studied the relationship among business model, big data, and enterprise innovation performance and found that big data technology can be employed as a driving force for enterprise innovation and development [13].

In the above research on enterprise business model innovation, the research direction is mostly the macro research on the whole business model innovation, so the research results are more general, and the research on Internet enterprises is less. Hence, the decision-making field, one of the components of the business model, is selected for research and analysis. Game theory and neural network models are introduced to innovate in the field of decision-making under big data.

Game theory, which was put forward in the 1840s, is a theory to study the rational decision-making behavior of decision-makers and the equilibrium of decision-making results, which interact and depend on each other. It is mainly adopted in economic analysis and has been applied in many fields. The game theory highlights the concept of rationality. Coelho and Sandes put forward the concept of “solution.” The importance of individual rationality in the game is evaluated through the analysis of the game results [14]. Lv et al. pointed out that rational factors should be combined with irrational factors. Game theory plays an extremely crucial role in breaking the oligopoly of enterprises [15]. The neural network began to develop in the 1960s and it has entered a high-speed development stage with the rapid development of computer technology. Karush and Rinki found that neural network has a strong interconnection, self-organization, adaptability, and learning ability [16]. Wang et al. showed that neural networks can effectively map functions [17]. Chang and Song studied the back-propagation neural network (BPNN) and found that BPNN greatly optimizes the problem-solving approach [18]. The game theory research method combining rational and irrational factors is selected and combined with the neural network model to analyze the problem.

To sum up, the business model innovation of Internet enterprises under big data is studied based on game theory and neural network model, and the research direction mainly focuses on enterprise decision-making. Models will be established for all internal and external decision-making of enterprises, including the market share neural model, the neural game model for oligopoly market decision-making, and model reflecting the decision-making relationship between managers and investors and between managers and employees. The research content provides a reference for the development of the neural network in an enterprise business model.

## 3. Model Construction Method of Business Model Innovation of Internet Enterprises

### 3.1. Influencing Factors and Foundation of Business Model Innovation Model

Market share is one of the crucial indicators to evaluate the performance of enterprises. The growth of market share is positively related to the improvement of return on investment and scale economy. Some studies have pointed out that the market share has a great relationship with the profit rate of enterprise investment. The accurate analysis of the changes in the market position of enterprises can be completed by comparing the data of market-leading enterprises with the market share of enterprises. The results lay a foundation for the innovation of the business model. However, many factors affect the market share. Thereby, it is essential to presuppose that there is no single company that can control the industry. Under this premise, the marketing effort of the market where the enterprise is located is directly proportional to the market share of the enterprise [19]. Some scholars have created relevant models to infer the market share of enterprises based on consumers' choice behavior and quantitative statistical method and analyze its attractiveness. However, these models have certain limitations and do not consider the restrictive factors of market share [20]. The influencing factors of market share are analyzed. Regarding the innovation of enterprise business model, first, the market share model combined with neural network is constructed to achieve the purpose of concise evaluation of the current business model.

The previous description shows that the market share of an enterprise is related to its marketing efforts and strategies. The elements of marketing include distribution strategy, price strategy, product strategy, and promotion strategy. The detailed data of these four parts are captured on the computer by using big data technology. The measurement of sales promotion and distribution is based on the support cost of enterprises for the two; the price is measured by statistical analysis of the score of product popularity; product information is scored 0–9 points based on consumers' choice. The higher the score is, the higher the product quality is. Finally, the score is counted.

The characteristics of oligopoly market include few manufacturers. There are only a few manufacturers in the market (when there are two manufacturers, we have what is called duopoly). Each manufacturer has a pivotal position in the market and has a considerable influence on its product price. These vendors are interdependent. When making decisions, any manufacturer must take into account the reactions of competitors, so it is neither the price maker nor the price receiver but the price seeker.. There is no difference in products, whether they are homogeneous or heterogeneous products, and the degree of interdependence is very high. It is called pure oligarchy. It is not easy to get in and out. It is quite difficult, even extremely difficult, for other manufacturers to enter. Other manufacturers are not only difficult to enter but also difficult to exit.

The control of the oligarchs in the industry is also a crucial factor of the enterprise market. Due to market restrictions, the product release of enterprises is subject to mutual restrictions. The participants of the game are all enterprises that put their own products in the market, but the number of products is limited. Hence, the total yield of *M* enterprises is set as *F* = *q*_1_ + *q*_2_ + … + *q*_*n*_. The relationship between the total selling price *p* and the total yield of the product is given based on previous research, as shown in the following equation:

(1) $$\begin{array}{c} p=p\left(F\right)=p\left[\sum_{i=1}^{M}p_{i}\right]. \end{array}$$

In (1), *F* is the total yield of the enterprise, and *M* is the total number of enterprises.

Zhu et al. proposed the importance of the relationship between enterprise managers and employees for enterprise development [21]. The decision-making model of managers and investors is constructed due to the crucial role of managers' decision-making in the business model. The relationship between managers and investors is determined by the contract signed by both sides, which is a kind of economic interest relationship. The contract is operable. Enterprise managers and investors supervise each other to achieve the purpose of common profit [22]. The employee is one of the crucial factors in business model innovation. Finally, the decision-making model between managers and employees is constructed [23]. The relationship between managers and employees is still contractual. Effective cooperation between managers and employees plays a positive role in the business model innovation. However, the contractual relationship between managers and employees is often incomplete, so it is easy to form a noncooperative game between them.

In conclusion, the market share model, the yield decision-making model of the oligopoly market, the decision-making model of managers and investors, and the decision-making model of managers and employees are constructed based on the neural network.

### 3.2. Establishment of the Market-Neural Network Model

The structure of BPNN is relatively simple. Its network training and learning are realized through the transmission error, and finally a certain expected output is obtained. The relationship among the influencing factors of market share is expressed based on neural networks.  Figure 1 displays the structure of BPNN.

Figure 1 suggests that the BPNN market share model is a three-layer structure. The research nodes include 1 output node, 4 input nodes, 1 middle layer, and 7 hidden layer nodes [24].

The working process of BPNN is expressed by equation. First, equation (2) is the concrete expression of the input of the hidden layer.

(2) $$\begin{array}{c} u_{j}=f\left(\sum_{i=1}^{n}O_{ij}x_{j}+\delta_{j}\right). \end{array}$$

In (2), *j* is the neuron of the hidden layer, *u* is the output value of the hidden layer, *x* is the input value of the hidden layer, *y* is the input neuron, *O* is the weight, and *δ* is the offset value of the hidden layer.

Equation (3) is the expression of the hidden layer and output layer.

(3) $$\begin{array}{c} y_{l}=f\left(\sum_{k=1}^{h}z_{lk}u_{k}+a_{l}\right), \end{array}$$

where *l* represents the neurons of the output layer (*l* = 1, 2,…, *m*), and *m* is the total number of neurons; *j* = 1, 2,…, *h*, and *h* is the total number of neurons. *z* is the output neuron, *v* is the weight, and *a* is the bias value of the output layer.

*f* in (2) and (3) represents the *S*-type growth curve function, and equation (4) shows its expression.

(4) $$\begin{array}{c} f\left(n\right)=\frac{1}{1+\exp\left(-n\right)}. \end{array}$$

In (4), *n* represents the part to be calculated in (2) and (3).

The core of BPNN is learning error, and equation (5) is the expression of learning error.

(5) $$\begin{array}{c} G=\frac{1}{2}\sum_{l=1}^{N}\overset{m}{\underset{i=1}{\sum }}\left(t_{l}^{i}-y_{l}^{i}\right). \end{array}$$

In equation (5), *G* is the learning error, *N* is the sample in the neural network, and *t* is the learning part. If the value of *G* is less than the known accuracy of the neural network, BPNN stops working.

The market-neural network model is constructed based on the above contents. First, the input and output of the learning samples are calculated, and then the bias value and weight of the neural network are modified. The two parts alternate until convergence occurs. The detailed network model construction steps are as follows.

First, the network state is initialized. Combined with the node number and the random number of the neural network designed in the previous sections, the bias value and weight of the network are set. Equations (6) and (7) are specific contents [25].

(6) $$\begin{array}{c} F_{7\times 4}^{1}\left(0\right)=\left[\begin{array}{cccc} 0.2 & 0.2 & 0.2 & 0.2\\ 0.2 & 0.2 & 0.2 & 0.2\\ \ldots & \ldots & \ldots & \ldots \\ 0.2 & 0.2 & 0.2 & 0.2 \end{array}\right],\\ a_{7\times l}^{1}\left(0\right)=\left[\begin{array}{c} 0.5\\ 0.5\\ 0.5\\ 0.5 \end{array}\right], \end{array}$$

(7) $$\begin{array}{c} F_{l\times 7}^{2}\left(0\right)=\left[\begin{array}{cccc} 0.2 & 0.2 & \ldots & 0.2 \end{array}\right],\\ a_{l\times 1}^{2}\left(0\right)=\left[0.5\right]. \end{array}$$

Equations (6) and (7) are the bias values and weights set for network initialization.

Then, learning mode *r*^0^ = *p*_*i*_·(*i* = 1) is input. The output of the hidden layer is obtained based on that (equations (8) and (9)).

(8) $$\begin{array}{c} r_{7\times l}^{1}=f^{1}\left(F_{7\times 4}^{1}r_{4\times 1}^{0}+a_{7\times 1}^{1}\right)=\log\text{sig}\left(F^{1}r^{0}+a^{1}\right), \end{array}$$

(9) $$\begin{array}{c} r_{l\times l}^{2}=f^{2}\left(F_{l\times 7}^{2}r_{7\times 1}^{1}+a_{l\times 1}^{2}\right)=\log\text{sig}\left(F^{2}r^{1}+a^{2}\right). \end{array}$$

Next, the learning error is obtained as follows:

(10) $$\begin{array}{c} e=g-r^{2}, \end{array}$$

where *g* is the expected output. Then, back-propagation is performed (equation (8)).

(11) $$\begin{array}{c} m^{2}=-2\left[f^{2}\left(n^{2}\right)\right]e. \end{array}$$

In (11), *n* is the number of pieces of data.

Finally, the BPNN gives the offset value and weight of the hidden layer, so the next input operation can be performed. The error is determined after the next learning model is input. When *i* > *n* and *e* > 0.01, the operation starts from the input of the learning model in the initial state again. Otherwise, it can be judged as the end of learning.

Lv et al. proposed the importance of simulation in machine learning [26], so simulation experiments are arranged. The market share of a well-known Internet enterprise is taken as an example and analyzed. First, the basic information of 6 products in the enterprise is collected by the literature method, and the share of 6 products is analyzed and compared. Then, the designed market-neural network model is employed to obtain the threshold and weight of each node, and the accuracy of the results is verified. If the accuracy is higher than 90%, it is excellent. Finally, the solution strategy is studied, and the original scheme of increasing market share is improved. The improved scheme is assumed and input into the market-neural network model for simulation experiment, and the product optimization scheme is obtained.

### 3.3. Construction of Yield Decision-Making Model in the Oligopoly Market

#### 3.3.1. Yield-Price Relationship Model

The total yield of the market in which the enterprise is located affects the price at which all products are sold. Besides, the market environment, national policy, and season also exert an impact on product prices. Experts are consulted to score since many influencing factors cannot be quantified.  Figure 2 presents the neural network structure of the yield-price relationship.

Figure 2 reveals that the structure of the neural network model of yield-price relationship consists of two parts: the relationship between yield and price and the relationship between price and various influencing factors simulated by BPNN algorithm. *F* is the linear relationship between yield and price: *F* = *r*−Af. *r* and *a* are influence factor constants, which need to be trained by neural network model.

As the structure of the neural network model here is consistent with that of the market-neural network model mentioned above, the overall equation expression and process of the neural network will not be repeated here. The expression of the relationship between yield and price in the final neural network based on previous studies is given as follows:

(12) $$\begin{array}{c} q=\frac{f}{d}-\frac{1}{d}F. \end{array}$$

In (12), *q* is the price, and *F* is the yield. *f* and *d* are the parameters of the neural network model.

#### 3.3.2. Enterprise Decision-Making Model

The enterprise decision-making model is based on equation (12) and game theory. First, equation (13) is the expression of enterprise profit:

(13) $$\begin{array}{c} T_{i}=f_{i}\times q\left[\sum_{i=1}^{n}q_{i}\right]-f_{i}c_{i}-\lambda c_{i}f_{i}=f_{i}\left[q\left[\sum_{i=1}^{n}q_{i}\right]-c_{i}\right]-\lambda_{i}c_{i}f_{i}. \end{array}$$

In (13), *c* is the marginal production cost, and *λ* is the risk index.

Equation (14) can be obtained by transforming equation (13) into yield reaction function.

(14) $$\begin{array}{c} f_{i}=R_{i}\left(f_{1},\ldots ,f_{n}\right)=\frac{1}{2a}\left[r-\left(1+\lambda_{1}\right)c_{i}\right]-a\sum_{j=1}^{M}f_{i}. \end{array}$$

When there are *M* enterprises, *n* reaction functions can be combined to get the profit function, as shown in the following equation:

(15) $$\begin{array}{c} T_{i}=\frac{1}{a}{\left[\frac{1}{M+1}\left(r+\sum_{i=1}^{M}\left(1+\lambda_{1}\right)c_{i}\right)-\left(1+\lambda_{1}\right)c_{i}\right]}^{2}. \end{array}$$

The profit functions of *M* enterprises are input into the neural network, and the results are compared. The data of 10 Internet enterprises are selected for comparative analysis.

Next, the enterprise cooperation decision is analyzed. Enterprises will cooperate and monopolize production in order to maximize their profits when they choose to cooperate. Equation (16) is the profit function of all manufacturers in this case.

(16) $$\begin{array}{c} T=\text{rnf}-{\text{aM}}^{2}f^{2}-f\sum_{i=1}^{M}\left(1+\lambda_{1}\right)c_{i}. \end{array}$$

The solution is obtained from the data of the enterprise, as shown in the following equation:

(17) $$\begin{array}{c} T_{i}=\frac{1}{a}\left[\frac{rM+\sum_{i=1}^{M}\left(1+\lambda_{1}\right)c_{i}}{2M}-\left(1+\lambda_{1}\right)c_{i}\right]\times {\left[\frac{\text{rM}-\sum_{i=1}^{M}\left(1+\lambda_{1}\right)c_{i}}{2{\text{aM}}^{2}}\right]}^{2}. \end{array}$$

Finally, this equation is substituted into the neural network model to compare the profits of enterprises.

#### 3.3.3. Decision-Making Model of Enterprises Seizing Market

The phenomenon of seizing the market in enterprise competition is studied, which is characterized by the profit function after seizing the market. Equation (18) is the profit function of an enterprise after seizing the market.

(18) $$\begin{array}{c} f_{i}=\frac{1}{2a}\left[r-\text{Mc}+\sum_{i=2}^{M}c_{i}\right],\\ T_{i}=\frac{1}{4\text{aM}}{\left[r-\text{Mc}+\sum_{i=2}^{M}c_{i}\right]}^{2}. \end{array}$$

Equation (19) is the profit function of the following enterprises.

(19) $$\begin{array}{c} T_{i}=f_{i}\left[r-c_{i}-a\sum_{i=1}^{M}f_{i}-\frac{r-\text{Mc}+\sum_{i=2}^{M}c_{i}}{2a}\right]-c_{i}f_{i}. \end{array}$$

The yield and profit of the following enterprises are obtained after equation (19) is derived, as shown in the following equation:

(20) $$\begin{array}{c} f_{i}=\frac{1}{a}\left[\frac{1}{2M}\left[r+\text{Mc}+\sum_{i=2}^{M}c_{i}\right]-c_{i}\right],\\ T_{i}=\frac{1}{4\text{aM}\times M}\left[r+\text{Mc}-2c_{i}-\sum_{i=2}^{M}c_{i}\right]. \end{array}$$

An enterprise that grabs the market and five following enterprises are selected to compare their yield and profit.

### 3.4. Construction of Decision-Making Model of Managers and Investors

Due to the contractual relationship between managers and investors, they check and balance each other and play a dynamic game to achieve the purpose of mutual supervision.  Figure 3 shows a game model.

Figure 3 shows that the manager-investor game model consists of three parts. After investors make a choice, managers decide whether to accept or not, and finally managers decide whether to work hard.

Managers and investors enter into the game stage after signing the contract. Managers choose to work hard or be lazy and take risks, while investors choose to pay more or pay nothing and take consequences. 10 Internet companies are selected to obtain their data and combined with the model to compare the relationship between managers' efforts and results.

### 3.5. Decision-Making Model of Managers and Employees

The relationship between the decision-making of enterprise managers and employees is studied from the conflict between them. In general, there is an appropriate wage level to ease the conflict between managers and employees. The level of wages affects the attitude of employees and the cost of enterprises, so there is a game between managers and employees. The employee chooses or does not choose the salary and treatment given by the manager. Once accepted, employees can choose hard work or slack work, and managers will choose whether to continue to cooperate when they find their slack behavior.  Table 1 displays the specific content of the game.

In Table 1, pR−h represents the manager's expected return. The game strategy is analyzed based on Table 1. Equation (21) presents the profit of employees under the condition of hard work.

(21) $$\begin{array}{c} v=\frac{h-g}{1-\vartheta }. \end{array}$$

*φ* represents the discount factor.

The profit situation of employees under different conditions is compared based on equation (12).

## 4. Analysis on the Results of Internet Business Model Innovation Model

### 4.1. Results Analysis of the Market-Neural Network Model

Internet products are divided into *C*-end products, *b*-end products, data and strategy products, commercial realization products, and AI products. From the perspective of target users alone, data and policy products may be *b*-end products or *C*-end products. However, due to the strong relevant professional knowledge required to be responsible for data and strategy products, in practice, it is not the responsibility of ordinary product managers but the responsibility of special data and strategy product managers. 6 products of Internet enterprises are selected to analyze and compare their market share.  Figure 4 shows the result.

Figure 4 shows that, among the products of the 6 enterprises, product no. 1 has the highest market share (36.1%), and its brand popularity is also the highest (9 points). However, its product price, product quality, and distributor fees are not the highest. Product no. 2 ranks second in the market share, with good quality, 8 points of brand popularity, and the highest distributor fee of 2.3 yuan. The product with the smallest market share is product no. 6, with a market share of 3.1%. Its product price is in the middle level, but the brand popularity is the least. The data analysis shows that the market share of a product is most affected by the brand popularity, followed by the product quality, and the market share is less affected by the product price and the distributor fees. The market share of the product 3 is in the middle position, and it is easy to become a follower in the market, but the marketing strategy of the product needs to be changed in order to improve the market share.

Moreover, the designed market-neural network model is adopted to obtain the threshold and weight of each node.  Figure 5 displays the result of obtaining the accuracy.

Figure 5 illustrates that the accuracy of the designed market share neural network model reaches 93% at the highest level and 89% at the lowest level. The reason may be that the network training of hidden nodes is incomplete. However, the overall accuracy level is qualified, indicating that the model is feasible.

Finally, the solution strategy is studied. Product no. 3 in Figure 1 is studied, and Figure 6 is a comparison of the optimization schemes of the product.

Figure 6 suggests that the market share of scheme no. 4 is the highest, reaching 39.5%. This is because scheme no. 4 is to adjust the brand popularity of the original scheme to the highest level, improve the product quality to 4.5, and increase the distributor fees. However, scheme no. 4 requires enterprises to become leaders and challengers in the industry. Schemes no. 1, no. 2, no. 3, and no. 5 have a small increase in market share, which is due to the lack of brand popularity, that is, no commercial marketing. The last scheme is to strengthen the market thrust of the product, and the market share of the product has also been significantly improved. It indicates that not only can the improvement of market share rely on price reduction but also it needs to improve the profit of distributors and improve the brand image.

### 4.2. Construction of Yield Decision-Making Model in Oligopoly Market

#### 4.2.1. Result Analysis of Enterprise Decision-Making Model

The independent decision-making data and cooperative decision-making data of 6 Internet enterprises are selected for comparative analysis, mainly for the analysis of yield and profit.  Figure 7 displays the comparison results.

Figure 7 displays that when the 6 enterprises make independent decisions, the maximum yield is 1934 pieces, the minimum yield is 1178 pieces, the maximum profit is 119 yuan, and the minimum profit is 92 yuan. When the 6 enterprises make the cooperative decision, the yield of the enterprise reaches 4433 pieces, and the enterprise gains 1825 yuan. It reveals that a cooperative game is the best choice. Enterprises need to unite to find the best way to benefit, instead of only considering their own interests.

#### 4.2.2. Analysis of the Results of the Decision-Making Model for Enterprises to Seize the Market

An enterprise that seizes the market and five following enterprises are selected to compare their yield and profit.  Figure 8 displays the comparison results.

Figure 8 suggests that the market leader's yield and profit are the largest, reaching 17672 pieces with a profit of 10106 yuan. The yield and profit of followers in the market are much less, with a minimum of 2443 pieces and a profit of 599 yuan. The leader in the market gets the biggest profit, but it is easy for the leader to limit production and bid, which makes it fall into the dilemma of constant competition but extremely low profit. Enterprises should choose to cooperate to maintain healthy competition.

### 4.3. Construction of Decision-Making Model of Managers and Investors

6 Internet companies are selected to obtain their data and combined with the model to compare the relationship between managers' efforts and results. Score comparison is used.  Figure 9 presents the comparison results.

Figure 9 suggests that there is a positive correlation between the efforts of managers and the results obtained. The basic wage of managers is the highest (3500 yuan) when their effort degree reaches 30. When the effort degree of managers is 9, the basic wage and share are the lowest, which are 1000 yuan and 7.5%, respectively. It reveals that the higher the effort degree of managers is, the higher the results will be. However, the basic wage of managers does not increase further after the effort degree of managers reaches 35. The reason is that the effort limit of managers is about 35.

### 4.4. Construction of Decision-Making Model of Managers and Employees

In the decision-making model of managers and employees, 6 employees with different basic wages in an Internet enterprise are selected to compare the relationship between their wages and efforts.  Figure 10 shows the comparison results.

Figure 10 displays that there is a positive correlation between the level of work effort and the basic wage. The basic wage reaches the highest value (1500 yuan) when the employee's effort degree is 40. It is 500 yuan when the employee's effort degree is 15. Moreover, the basic wage will not increase when the effort degree reaches 50. It is speculated that 50 is the effort limit of Internet employees. Combined with the previous content, it is obvious that managers will continue to hire employees with higher effort degrees.

## 5. Conclusion

Based on game theory and neural network model, this paper studies the business model innovation of Internet enterprises under big data, and the research direction mainly focuses on enterprise decision-making. It will establish models for all internal and external decisions of enterprises, including market share neural model, oligopoly market decision-making neural game model, and model reflecting the decision-making relationship between managers and investors and that between managers and employees. This exploration is to study the business model innovation of Internet enterprises with the decision-making field as the breakthrough point. Game theory is combined with neural networks to discuss the business model innovation under the background of big data. The results show that different decisions exert different effects on the development of the business model. The research content provides a new reference path for the innovation of the enterprise business model. However, there are still some deficiencies. In the discussion of decision-making for managers, the research is not deep enough. The influence of other external factors, such as the rise and fall of market economy and financial crisis, needs further verification. In the future, in-depth research can be conducted on this part to make the research conclusion more convincing.

## Figures and Tables

**Figure 1:** BPNN market share model.

**Figure 2:** Neural network structure of yield-price relationship.

**Figure 3:** Manager-investor game model.

**Figure 4:** Sample data of market share of a product.

**Figure 5:** Accuracy rate of the market-neural network model for a market share of a product.

**Figure 6:** Comparison of product optimization schemes.

**Figure 7:** Comparison of enterprise decision-making under the yield decision-making model of oligopoly market.

**Figure 8:** Comparison of yield and profit under the decision-making model of enterprises seizing the market.

**Figure 9:** The relationship between manager's effort and results under the decision-making model of managers and investors.

**Figure 10:** The relationship between different basic wages and effort of employees.

**Table 1:** Manager-employee game.

Personnel category	Employee		
Manager		Slack	Strive
	Hire	*R*−*h*, *h* − *g*	pR−*h*, *h*
	Do not hire	0, *h*_0_	0, *h*_0_

Note: *R* is the income, *P* is the probability of occurrence, *h* is the employee's wage, and *g*is the utility loss caused by labor.

## Data Availability

The data used to support the findings of this study are available from the corresponding author upon request.
